The article "Study on Coupling Coordination Degree between Regional Sports Industry Development and Healthy China Construction" was published in 2022. Journal: J Healthc Eng.

# Study on Coupling Coordination Degree between Regional Sports Industry Development and Healthy China Construction

**DOI:** 10.1155/2022/7785267

**Published:** 2022-02-07

**Authors:** Li Tang

**Affiliations:** The Engineering &Technical College of Chengdu University of Technology, Leshan, Sichuan 614000, China

## Abstract

“Healthy China” is one of the most important goals in the development of China's sports industry, which contributes to the realization of the macro development strategy of “Healthy China” and becomes the main trend of supply-side reform of sports industry. The realization of a healthy China can not be separated from the development of sports industry, and we can see that the future development of sports industry will have great prospects. The innovative development of sports industry economy not only shows the characteristics of the times, but also is a brand-new economic format from the perspective of public concern. The development of sports industry plays a fundamental role in the process of building a healthy China. By providing diversified and multi-level sports products and services, it can enhance the health value, enrich the healthy life and increase the healthy experience of consumers, thus promoting the building of a healthy China. This paper starts with the analysis of the opportunities of sports industry development under the healthy China strategy, and analyzes the implementation strategies of sports industry economic innovation and development under the healthy China strategy.

## 1. Introduction

Health is an inevitable requirement to promote people's all-round development, a basic condition for economic and social development, an important symbol of national prosperity and national prosperity, and a common pursuit of the broad masses of the people [1]. Then, under the background of healthy China's macro development, how to optimize the supply-side reform of sports industry has become a critical development issue [2]. Man is the subject of social development and the ultimate goal of social development. Health is an eternal topic pursued by human generations. The level of health affects people's quality of life, as well as the fate of the country and the rise and fall of the nation [3]. At present, driven by society and government, health industry has become a new driving force for global economic development. Vigorously developing regional sports modernization is an important core content of China's regional coordinated development, which is also consistent with the implementation of industrial development, ecological civilization, social stability, healthy life and other modern urban and rural overall construction in the national overall development plan [4]. The 19th National Congress of the Communist Party of China put forward the implementation of Rural Revitalization Strategy, which reflects the development requirements of China's current modernization construction and changes in urban-rural relations, and is the fundamental task of building a moderately prosperous society in an all-round way [5]. Accelerating the construction of healthy China and consolidating the healthy cornerstone of building a moderately prosperous society in an all-round way has become an important strategic goal and policy proposition in China's great journey in the new era [6]. With the increasingly prominent role of digital technology in promoting China's sports industry, digitization in the field of sports industry points out the breakthrough direction and path for the development of new formats. According to Jiang Xiaojuan, Professor of the school of public management of Tsinghua University, with the support of technologies and industries such as 5 g, artificial intelligence, big data, cloud computing, Internet of things and various intelligent device manufacturing, sports digitization will develop rapidly along the two paths of “digital technology + industry” and “traditional industry + digital technology”, and become the main growth point of the development of sports industry.

Physical exercise is one of the ways to implement healthy China. At present, most people prefer to play with electronic products at home. Only a small number of people will choose physical exercise to enrich their leisure time, resulting in the poor physical quality of most people [7]. Healthy China is not only a new development concept, but also a goal based on the reality of the masses, and a blueprint for the development of a well-off society in an all-round way [8]. Therefore, under this strategic requirement, we must pay full attention to the factors affecting public health, and on this basis, formulate scientific and reasonable industrial development strategies, and build a new mechanism for the economic innovation and development of sports industry [9]. The construction of healthy China is a systematic project and a blueprint for national health under the background of building a moderately prosperous society in an all-round way. As an important part of the national economy, sports industry is becoming an important force in China's economic restructuring, transformation and upgrading, employment security and innovation driven under the new normal [10]. Starting from the analysis of the opportunities of the times for the development of sports industry under the healthy China strategy, combined with the current problems in the process of economic development of China's sports industry, this paper analyzes the implementation strategies for the economic innovation and development of sports industry under the healthy China strategy.

This paper is divided into four parts. The first part needs to elaborate the research background of healthy China. The second part expounds the opportunities for the economic development of sports industry under the strategy of “healthy China”. This paper expounds that people should pay attention to health and improve the concept of development. The third part studies the economic innovation and sports industry development strategy under the “healthy China” strategy, integrates resources and creativity, improves policies and increases investment. Finally, the full text is summarized.

## 2. Opportunities of the times for the Economic Development of Sports Industry under the Strategy of “Healthy China”

### 2.1. Focus on Health

Sports industry is an extremely important industrial form in China's national economy, and its value is extremely diversified during the development of sports industry. Economic value and cultural value are both important components of its value. In the development of China's social sports, the regional public sports service system plays an important leading role, leading the development direction of China's mass sports, and effectively matching the fitness and leisure sports industry with the public sports service system is an important driving force for the strategic development of “Healthy China”. Sports services are listed as an important part of health promotion services, and sports fitness and leisure, sports training, sports rehabilitation, and stadium services become the main body of integration. What is interpreted behind the good and systematic sports industry is a series of sports-related industrial mechanisms, such as sports event economy, sports insurance, sports tourism and so on. At the same time, the mature and systematic sports industry economy is also enlightening and guiding the public to participate widely. In this process, it effectively meets the public's fitness demands, thus creating a cultural atmosphere for the public to actively exercise [11]. The products and services provided by the sports industry are characterized by functional prevention, high elasticity of demand and comprehensive benefits, which are mainly “preventing diseases”. They are a more active, more profitable and longer-term health investment way than medical services, and can maintain and promote physical health in the whole life cycle.  Table 1, for example, is a survey of the desire rate in the sub-key period of leisure sports guidance.

The structural adjustment of sports industry is carried out from the angle of actual demand, and sports consumption demand is fully stimulated by sports supply. In this process, public sports service affects the development quality and level of sports industry to a certain extent. Based on the health concept of whole-course intervention, combined with the application of big data and sports medical technology, sports fitness service provides scientific and systematic solutions such as sports health consultation, physical fitness test, sports health assessment, sports guidance, health advice or early warning, and meets the needs of fitness shaping, sports and health care, thus becoming an effective means to prevent and treat chronic diseases and alleviate sub-health status. Today, with the increasing demands of the public for health, the advantages and influence of the sports industry have become increasingly prominent. Sports is a non-medical way of health. To a certain extent, scientific and systematic sports can effectively make up for the deficiency of medical care in maintaining public health activities [12].

### 2.2. Upgrade of Development Concept

Sports industry is an industry of people's livelihood and happiness, which plays an irreplaceable role in meeting people's growing needs for a better life. With the in-depth development of sports industry, people's health awareness gradually awakens, paying more and more attention to the healthy quality of life, and sports consumers such as sports fitness and sports tourism are increasing. Regional sports industry; economic development Abstract: regional economic integration is one of the most striking economic phenomena in current international economic relations. It can be the formation of multi-national regional economic integration or different administrative regions within a country. Regional sports industry integration is the rudiment of developing sports industry base system. Sports industries that provide sports products and services to the society will form an integrated sports industry base through integration and development. The diversification of elements in the system can quickly improve the energy efficiency of industrial development and enhance its core competitiveness. Promoting supply-side structural reform is a major innovation to adapt to and lead the new normal of economic development, and it is the breakthrough and focus of China's economic transformation and upgrading.

Deepening the supply-side structural reform, innovating the transformation and upgrading of sports industry, promoting regional cooperation and forming the integration of sports industry are new opportunities for the integration and development of regional public sports services and local sports industries.  Figure 1 is the development model of urban agglomeration.

Following the laws of market economy, the sports industry adopts commercial operation mode to allocate sports resources in a market-oriented way. By creating splendid sports events, sports tourism, sports fitness services, sports culture fairs and other product systems, sports cultural resources can be developed more effectively, sports cultural charm can be displayed, and a healthy cultural atmosphere can be created. The guiding structure of strategic adjustment of urban industrial structure is shown in Figure 2.

Faced with the huge demands of the public for fitness, the sports industry can give full play to a series of development advantages such as numerous projects, broad mass base and profound influence, and optimize the industrial development concept by integrating various resources in the whole industry, so as to truly meet the public's enthusiasm for fitness and their demand for health. In terms of demand structure. There is a seesaw relationship between medical health demand and non-medical health demand. The stronger the non-medical health demand is, the more rational the demand structure of health industry is. Under normal circumstances, the more non-medical health needs, the less medical health needs. At this time, the better the health status of residents, the corresponding reduction in medical expenses. Nowadays, people's pursuit of health is no longer a kind of exercise and fitness, but a positive and optimistic way of life. Therefore, all kinds of healthy contents can be integrated into the industry, and both tangible products and intangible services can become important elements of the development of the industry.

## 3. Economic Innovation and Development Strategy of Sports Industry under the Strategy of “Healthy China”

### 3.1. Integrating Resources and Creativity

Sports industry economy is a relatively independent industrial form with rich connotations. Under the influence of the healthy China strategy, national fitness has gradually developed into a social trend. The promotion of this strategy aims to enable the whole public to form a healthy and optimistic state of mind and body, and effectively improve the public's happiness. With the improvement of income level, people's life style has changed greatly, service consumption and non-material consumption will increase explosively, and the proportion of sports consumption in family life consumption is getting higher and higher. Constructing cooperative supply mechanism is an inevitable choice for the coordinated and benign development of sports industry and public sports services. In the report of the 19th National Congress of the Communist Party of China, it is pointed out that social organizations, as important social forces, should give full play to the role of public service supply. To a certain extent, the collaborative supply mechanism of public services is an effective judgment of public service supply from the perspective of satisfying the pursuit of happy life by social members.

In the process of economic development of sports industry, we should deepen the market-oriented reform and speed up the diversified layout of sports industry by perfecting the development policies of sports industry.  Table 2 lists the reasons for not wanting to engage in sports activities and the problems that must be solved when participating in sports activities.

With the increasing development of the current sports industry market, the government should nurture a group of sports enterprises and brands with great development advantages through policy guidance and fiscal tilt, and improve their professionalism through market-oriented operation. The integration mechanism of public sports service and local sports industry refers to the processing mode of various elements in the process of promoting the integration of sports industry by public sports service. In the process of integration and development, it needs to rely on the joint action of internal power and external power. In the process of controlling service quality and promoting the development of sports industry, it needs evaluation, supervision and guarantee mechanism to participate in the operation.

### 3.2. Improve Policies and Increase Investment

Stimulated by a series of factors, such as industrial structure adjustment, healthy China strategy and promotion of sports consumption, the future sports industry will inevitably develop in the direction of diversified formats, multi-modal consumption and high quality. Especially, driven by the concept of sharing and “Internet plus,” the integration between industries is deepening, and the integration between sports, tourism, culture and commerce is increasing day by day. “Sports+” has become an agglomeration advantage. In the process of the integration of public sports service and sports industry, it is an important guarantee to establish the information feedback mechanism of public sports service demand expression and adjust the direction in time by analyzing and summarizing the feedback information, which is to realize the high efficiency, sharing and sustainable innovation development of the integrated operation mechanism of regional sports public service. Combining the development planning of the whole city sports industry with the development planning of public sports facilities, and fully considering the saturation of sports space that the city can achieve, it is also the development planning of public sports facilities designed based on people's livelihood sports demands. The government should give full play to its leading position in the economic development of sports industry, and realize the value of “healthy China” by reasonably defining the responsibilities of all parties and maintaining the order of sports market. First, take the sports department as the main body, deeply integrate healthy China with the construction of the whole people, and fully integrate sports health with medical health, so as to realize the era pattern of “great health”.

## 4. Conclusions

With the increasing emphasis on sports in China in recent years, the innovative development of sports industry plays an increasingly prominent role in promoting the implementation of the development strategy of a sports power. Public sports service is a safeguard measure derived from the development of social economy to a certain extent, which helps to enhance the economic effect of sports industry. Sports industry, as the industry most closely related to the concept of healthy China, will be deeply influenced by healthy China. The proposal of “Healthy China” has brought great opportunities and challenges to China's sports industry, which not only promotes the development of sports industry, but also brings certain challenges to related talents in sports industry. With the development of healthy China strategy, sports industry has also developed into the “new darling” of public life. Therefore, taking the concept of “industrial economy” as the breakthrough point, exploring the specific strategies of economic innovation and development of sports industry will not only directly affect the goal of national fitness, but also be the firm cornerstone for realizing the goal of “healthy China”. Nowadays, people's pursuit of health is no longer a kind of exercise and fitness, but a positive and optimistic way of life. Therefore, all kinds of healthy contents can be integrated into the industry, and both tangible products and intangible services can become important elements of the development of the industry. However, this study also needs to further promote the development of China's sports industry health strategy. Public sports service is a safeguard measure derived from social and economic development to a certain extent. Therefore, in the future research, it is also necessary to conduct in-depth research on public health.

## Figures and Tables

**Figure 1:** Development model of urban agglomeration.

**Figure 2:** Strategic adjustment guide structure of urban industrial structure.

**Table 1:** Survey on the sub-period desire rate of leisure sports instruction.

Option	Frequency	Preface
Establish community sports facilities	65.1	1
Open sports venues	43.4	2
Have someone to guide physical exercise	42.4	3
Strengthen the propaganda of sports knowledge and exercise methods	30.5	4

**Table 2:** Ranking survey results.

Reasons for unwillingness to engage in sports activities	There are no sports facilities	Heavy work, physical and mental fatigue	Don't know how to exercise	Not interested	Insufficient economic strength
Problems that must be solved in participating in sports activities	There are venues and equipment	With guidance	Have economic conditions	With companions	Overcome inertia
Sort	1	2	3	4	5

## Data Availability

The data used to support the findings of this study are included within the article.

## References

[1] Xin C., Liping L. (2017). Opportunities and challenges of the sports leisure industry under the healthy China strategy. *Contemporary Sports Science and Technology*.

[2] Huijuan S., Jieyou Z., Xiukuan G. (2021). The main problems, causes and solutions in the field of fitness and leisure industry in China. *International Journal of Sports Science and Physical Education*.

[3] Bo L. (2018). The development of traditional national sports industry under the background of healthy China. *Value Engineering*.

[4] Yu Y. (2019). Theoretical explanation and policy thinking of “national fitness” and “healthy China”. *Journal of Beijing Sport University*.

[5] Li S., Wu X., Yang S. (2018). Discussion on several issues of sports consumption upgrade under the background of “healthy China”. *Sports Boutique*.

[6] Li J., Kim S. Y. (2019). On the development direction and policy of Chinese school physical education under the background of healthy China 2030 program. *International Journal of Emerging Multidisciplinary Research*.

[7] Zhang Y., Zhang B., Du H., Xu C. (2018). Research on the path of creating sports towns under the background of “healthy China”. *Journal of Harbin Institute of Physical Education*.

[8] Zhao L., Li J. (2017). Analysis of obstacles to the improvement of the competitiveness of my country’s leisure sports industry. *Journal of Shenyang Institute of Physical Education*.

[9] Song F. (2019). Research on the curriculum setting of “integration of sports and medicine” in sports colleges under the background of “healthy China. *Contemporary Sports Science and Technology*.

[10] Ren B. (2020). Dynamic measurement research on the interactive relationship between China’s sports industry and cultural industry. *Sports Research*.

[11] Woźniak M. G. (2019). Integrated development and modernisation of human capital are needed. *Nierówności Społeczne a Wzrost Gospodarczy*.

[12] Zhu J. (2018). Value analysis and development path of sports towns from the perspective of global tourism. *Sports Research and Education*.

